# Research on  Making  Use of  Sports Tourism Resources to Build and Develop Sports Leisure Towns (Small Towns in Guangxi)

This article has been retracted.

**DOI:** 10.1155/2022/2801232

**Published:** 2022-07-18

**Authors:** Jucheng Yu, Xiaohua Ma

**Affiliations:** ^1^Nanning University, Nanning, Guangxi 530200, China; ^2^Hezhou University, Hezhou, Guangxi 542899, China

## Abstract

With the continuous progress of the times, people's economic level has also improved, and they have more specific requirements for their own quality of life. At present, looking at the domestic health industry, its development is far from meeting people's expectations. In recent years, the state has advocated the construction of a number of sports characteristic small towns with national participation, beautiful ecology, industrial integration, and distinctive characteristics. The Guangxi government responded to the national initiative and actively supported it in policy, introduced investment funds, and established eight sports characteristic small towns, which are in good condition of development. This study takes this as the research object, through consulting various literatures, data material, and visiting experts and scholars, actually checks the development of these eight characteristic small towns, and sorts out and analyzes the collected information on its natural resources, humanistic characteristics, and diversified industrial integration. It provides a theoretical basis for the subsequent design, planning, and practice of characteristic small town. After the overall normative construction and taking the normative effect as the empirical evaluation standard, it has effectively promoted the vigorous development of small towns with sports characteristics in China.

## 1. Introduction

Due to the continuous progress of economy and society, people's requirements for a healthy life have increased. In 2017, China's General Administration of Sports issued a notice on promoting the construction of sports and leisure characteristic small town. In the document, people's governments across the country are encouraged to establish a number of national sports activities in which local people's governments all over the country are encouraged to build up a number of cities dominated by national sports activities, with superior natural environmental conditions and green sports small town with strong historical and cultural characteristics. Therefore, Guangxi province a large number of sports characteristic small town have been built throughout the province. In the same year, the people's Government of Guangxi Province issued the “Healthy Guangxi 2030 Plan,” which proposed to build a healthy rural demonstration area, a leisure and fitness farm demonstration park, and a fruit display industry base [1]. Small town built up with sports characteristics in domestic will become a new development direction of integrating urban and rural areas and integrating multiple business forms in China, which is bound to have a good development trend.

### 1.1. Research Purpose and Significance

This paper studies the development status and problems of characteristic towns based on sports and related industries after integrating the common development of many industries, including fitness service industry, leisure and health industry, and ecological environment industry. In addition, it explores a scientific and reasonable development path and promotes the rapid development of local economy and the future sustainable development of the townlet and its region [2]. This paper analyzes the deep meaning of building sports characteristic small town and constructs various types of models of sport characteristic towns so as to provide practical experience and strategic suggestions for the practice of “healthy Guangxi 2030.”

This study takes the development status of the small town as the research object, explores its construction in all aspects, establishes theoretical basis, and provides theoretical support and practical experience for the construction of characteristic small town in other cities. A small town with sports characteristics advocated by the state, supported by the government, and participated by capital will help the growth and development of local sports and related industries. Relying on the sports industry, when arousing people's love for physical exercise and promoting physical exercise for the whole people, the development of the town has practiced a new generation of national planning scheme for urban integration, accelerated the pace of economic development in the area where the characteristic town is located, and increased employment while arousing people's love for physical exercise projects and promoting physical exercise for the whole people. The local humanistic characteristics are publicized, people's awareness of protecting and loving the environment is enhanced, and theoretical basis and practical experience are provided for the subsequent establishment and implementation of characteristic small town. The specific meanings are as follows:

1. Lay the foundation for the sustainable future development of sports featured small town
2. Sound the discipline framework of scientific research in sports characteristic small town
3. Speed up the development rhythm of sports small town with sports characteristics in Guangxi and rely on the sports industry to drive the development of multiple industries
4. Improve the multilayer mix together development of Guangxi sports industry, carry out the construction of cities and towns integration, and promote economic development
5. Contribute to the strategic plan of “Healthy Guangxi 2030” and promote the integration of Health for All and Sports for all

### 1.2. Research Contents and Methods

#### 1.2.1. Research Contents

This paper takes eight sports characteristic small towns that have been completed and put into operation in Guangxi as the research object, compares the environmental advantages and development characteristics of each characteristic town, and analyzes its advantages and disadvantages in development [3]. Then, it explores the development status of various business forms of the characteristic town, explains the operation system of the town and the integrated application of various industrial resources, and analyzes and evaluates it. The list of the eight characteristic small towns is as follows: Mashan County sports characteristic town, beautiful southern sports characteristic town, Gayasi Valley sports characteristic town, Fangchenggang sports characteristic town, Chetian small township sports characteristic town, Lalang sports characteristic town, Xishanquan sports characteristic town, and Zhongdu Shili Luojiang sports characteristic town.

Firstly, this paper summarizes the overall development trend and local characteristics of the sports featured town. It studies the characteristics and shortcomings of the town. Then, it puts forward the conclusions and theoretical support with rationality, applicability, and long-term development (see Figure 1 for details).

#### 1.2.2. Research Methods

*(1) Documentation Method*. Search the relevant information, materials, policy document, and so on about “healthy China,” “healthy Guangxi 2030,” and “sports characteristic town” on the network. Carry out specific understanding and Research on the eight sports characteristic small towns in Guangxi so as to provide theoretical guidance for the follow-up development of the small town.

*(2) Field Interview Method*. In the process of this study, we specially visited the industrial operators, tourists, and local aborigines of the town, listened to practical experience and the real feelings of the masses, collected many different opinions and opinions on the construction of the town on the policy support and future development, and gathered the collected information of all parties.

## 2. The Empirical Research on the Development of Sports Characteristic Small Towns in Guangxi

Guangxi province, in response to the call of the state, takes the sports industry as the carrier to pilot establish a number of small towns with sports characteristics in the whole province. It is also an innovative practice policy in the planning of urban integration in the national policy [4]. Its small town is characterized by green health, ecological environmental protection, sports and leisure, and strong humanistic flavor. The advantage of the new development mode of small towns is that it cannot only promote the rapid economic development of small towns, but also promote the construction process of urban integration and the integrated development of multi-industries [5]. Guangxi General Administration of Sports has opened a green fast-tracked for engineering projects that apply for the construction of characteristic small town, stipulated the construction cycle for the successfully declared construction projects of small town, conducted a comprehensive investigation and evaluation after the completion of the construction cycle, and issued acceptance documents after passing the evaluation. The General Administration of Sports identified its construction project as “sports characteristic town.” See Table 1.

From the perspective of the main units applying for sports characteristic small town, most of them declaration subject are enterprises, there are few cooperation declarations between the government and enterprises. In terms of the declared industrial orientation, the project can be divided into natural type, national type and leisure type. (See Table 1 for details).

### 2.1. Natural Sports Characteristic Small Town

Natural type: it is a natural sports characteristic town with rich geographical environment and water resources. It is suitable for the development and utilization of sports projects and attracts tourists with its natural ecological resources, such as mountain shape and rivers, and environment [6]. Mashan county sports characteristic town, Chetian county sports characteristic town, and Lalang sports characteristic town are all sports characteristic small towns built on natural resources.

#### 2.1.1. Characteristic Townlet of Rock Climbing Sports in Guling Town, Mashan County

Mashan rock climbing sports characteristic town (as shown in Figure 2) is located in Mashan County, Nanning City, Guangxi Province, China, covering an area of 3.4 square kilometers. According to the urban area, it takes more than one hour by car and about two hours by bus. Relying on Nanning, the town has sufficient tourist resources. The county is surrounded by mountains, overlapping peaks, and obvious karst landform. The county is originally a poor area, but the natural scenery is pleasant and connected by mountains, which brings development opportunities for rock climbing.

The sports featured town in Mashan County is the first featured town with the theme of rock climbing in China. The small town has also built professional level tracks due to rock climbing projects. There are more than 500 tracks in total, many of which are natural rock wall tracks with high difficulty. Domestic professional rock-climbing teams also built training bases there, including the research and development of many rock-climbing tools and equipment also herein [7]. There are also rock climbing and mountain climbing outdoor training courses for children, teenagers, middle-aged, and elderly people, so they are favored by rock climbing enthusiasts of all ages and at home and abroad, which provide them with opportunities for exchange and learning.

The operation mode of the small towns is as follows: Sports + tourism + industry + events. The main regional planning includes four areas: rock climbing core area, rehabilitation and recreation area, business-supporting area, and hotel resort. This industrial layout scheme not only fully integrates the whole industrial chain, but also allows tourists to freely choose leisure and exercise methods. See Figure 2.

In a word, the town is in the stage of development and construction, and there are still many shortcomings. For example, during holidays and competitions, there are many athletes and tourists, but the number of professional coaches is insufficient, which increases the risk of sport. However, at ordinary times, there are few tourists and professional coaches are idle. The development prospect of the town is very good. We believe that through the honing of time and practice, the town will certainly develop its own business model and a first-class rock-climbing characteristic town in China and even in the world will be built [8].

#### 2.1.2. Chetian County Sport Characteristic Small Town, Ziyuan County, Guilin City

Guilin is a famous scenic spot in China, with magnificent natural landscape and rich experience in developing tourism industry. In recent years, Chetian county, a resource county under its jurisdiction, applied for a sports characteristic town project. Sport characteristic town is located in the southwest of resource county of Guilin city. It belongs to Miao village. It is rich in water resources, surrounded by mountains, and five rows of rivers flow through the town. The resources close to mountains and rivers have created favorable natural conditions for the development of sports characteristic small town.

The operation mode of the town is “sports + tourism + culture.” Taking Zijiang scenic spot as the carrier, it cooperates with the linkage development of famous scenic spots, such as Baoding Waterfall Scenic Spot, Bajiaozhai scenic spot, forest park, and Miao Yao ethnic scenic spot. Wupai river rafting is its core physical exercise project, which drives the surrounding outdoor cross-country, mountaineering, ecological expansion, and other sports, and focuses on building an “outdoor sports destination” [9]. New projects under construction in this town include Zijiang hot spring, resource snow scenery, and silver bamboo reserve.

The future development direction of the town lies in relying on holding sports events, combined with Miao characteristic sports programs and national customs and culture, to build a sports characteristic town with the common development of physical exercise, leisure and entertainment, and folk culture.

#### 2.1.3. Hechi Desheng Lalang Ecological Leisure Sports Characteristic Town

Lalang ecological sports characteristic town is located in Desheng Town, Hechi City, Guangxi, China, covering an area of 3000 mu. The town is built in Lalang ecological leisure tourism area. There are many famous scenic spots, such as forest farm and lake area and so on. The natural scenery is pleasant, the ecological environment is well protected, and the climate is like spring all the year round.

Relying on the Lalang leisure scenic spot, the town has been taking the forest farm as the core scenic spot for overall development and operation in conjunction with several other scenic spots in recent years. The built resort facilities include mountain climbing plank road, basketball court, forest animal and botanical garden, ecological corridor, and folk characteristic buildings. Because it has scenic spots as the carrier, it has rich operation and management experience and has a variety of entertainment facilities, such as leisure, vacation, accommodation, and catering. It often gives various entertainment programs, events, and competitions, such as concerts, bicycle events, color tune drama, dragon and lion performances, shadow boxing performances, horse riding, exploration, and so on [10]. Before applying for construction, it had held bicycle races relying on Lalang ecological leisure scenic spot. Now, it is expected to build a nearly 4 km long bicycle greening road. It is also the first four-star car tourism campsite in Guangxi Province, attracting many campers.

Since the beginning of operation, more than 50000 tourists have come to exercise and leisure vacation, and many enterprises and institutions have organized group construction, training, meetings, and so on. The town is building various ball games venues, pension centers, and other leisure facilities [11]. The operation mode of the town is as follows: Sports + ecology + tourism. The area is divided into cultural square area, various stadium areas, swimming area, and so on. The goal is to build a small town with sports characteristics integrating sports fitness, vacation and play, competitive events, and literary and artistic performances.

### 2.2. Ethnic Sports Characteristic Town

Ethnic type: ethnic-type small town with sports characteristics focuses on the original ethnic minority areas in small town and combines their traditional folk customs, unique cultural environment, and representative buildings as the basis for applying for small town with sports characteristics. Ethnic sports featured small towns include Gayasi Valley Sports featured town in Hechi Nandan and Zhongdu Shili Luojiang sports featured town in Luzhai county.

#### 2.2.1. Hechi South Dan Gayasi Valley Sports Characteristic Town

Hechi Nandan Gayasi Valley Sports characteristic town (Figure 3) is built in the Baiku Yao nationality spot of Nandan county. The natural environment in the scenic spot is pleasant and the ecological environment is well protected. The town covers a total area of 380 square kilometers. It is the residence of ethnic minorities, dominated by the living population of Baiku Yao nationality. Therefore, the sports programs held in the town have national characteristics, such as playing leather drums and going go up knife mountain. It is an area with well-preserved national physical exercise programs.

The operation mode of the town is as follows: Sports + tourism + folk custom. The regional planning is as follows: Car tourism camping area, sports park, core area, and poverty alleviation tourism area. The town has rock climbing facilities, kayaking competitive facilities, mazes, various ball facilities, as well as sports areas with strong national characteristics, such as bullfighting area, archery area, Hydrangea area, and other areas. The leisure area has anion fitness trails, health Tai Chi Valley, and so on [12]. The innovation of this town is to make use of the characteristics of ethnic minorities in the town to build a base with strong ethnic sports characteristics. While protecting and inheriting ethnic sports, it also drives the economic and social construction of ethnic areas, helps the communication between ethnic minorities, increases local employment opportunities, and creates jobs.

#### 2.2.2. Shili Luojiang Sports Characteristic Town, Zhongdu Town, Luzhai County, Liuzhou City

Shili Luojiang characteristic town in Zhongdu town is located in Luzhai County, Liuzhou. The small town has a history of more than 1700 years. It is a famous tourist town, close to Xiangqiao Karst National Geopark, a famous world geopark at home and abroad. It is the first batch of characteristic small town in China.

Since its establishment, the town has successively carried out many international sports, such as marathon, global cycling tour match, cross-country race, and so on. In combination with the development project of Zhongdu tourism area, various leisure and cultural facilities such as five-star leisure hotel, sports park, resort villa, health garden, and national museum will be built. Sports facilities include various ball venues, fitness trails, and bicycle trails [13]. The town is full of sports atmosphere and many people participate in the sports, which has laid a good foundation for the long-term development of the town.

### 2.3. Leisure Sports Town

A leisure town is one with comprehensive sports characteristics, with more diverse and modern entertainment and fitness equipment, and strives to create a rural environment for entertainment and relaxation. Leisure sports characteristic small towns include Xishanquan sports characteristic town, Fangchenggang sports characteristic town, and beautiful southern sports characteristic town.

#### 2.3.1. Guigang Guiping Xishanquan Sports Characteristic Town

Xishanquan is a small town with sports and cultural characteristics. It is located in Bailan village, Xishan County, Guiping, China, covering an area of about 30 square kilometers. It is close to the mountain and water, with a good natural environment. There are many world-famous natural scenic spots nearby, such as Longtan National Forest Park, Jintian uprising old residence scenic spot, and so on, relying on the hot spring health preservation resource area. It has held many events, such as camping festival, tourism festivals, art festivals, food festivals, ethnic minority activity festivals, and so on. The operation mode of the town is as follows: Sports + tourism + health preservation, which is divided into sports area, leisure area, cultural expo area, health preservation area, hot spring area, and business area. The town integrates ecological health preservation, sports, elderly care, and leisure, focuses on sports and cultural health preservation, and attracts many tourists to experience and play.

#### 2.3.2. Fangchenggang Sports Characteristic Town, China

Fangchenggang sports characteristic town (Figure 4), located in the middle and lower parts of Guangxi, is a small seaside town in China's coastal areas, with good advantages in water resources. Relying on coastal natural resources, it has developed many water sports such as sailing, water motorboat, and surfing, and has held China ASEAN marathon, world-class bicycle tour, cross-country challenge, sailing, and so on [14]. These events not only brought tourists and resources to the town, but also established a platform for mutual communication between China and ASEAN countries.

The operation mode of the town is as follows: Sports + events + industrial integration. The area is divided into business meeting area, entertainment business area, mountain sports area, medical and health area, water sports area, and other activity areas. In the town, leisure, entertainment, and sports projects drive the development of relevant catering and accommodation industries and build an ecological chain system of joint development of multiple industries based on small towns.

#### 2.3.3. Beautiful Southern Cycling Sports Characteristic Town

Located in Xi Xiang Tang District, Nanning City, Guangxi Province, China, the beautiful southern sports characteristic town is called the urban back garden of Nanning city because of its picturesque scenery. In addition to the unique leisure and vacation ecosystem, there are also a variety of industries integrated in the town, such as health preservation area, sports area, cotton craftsman garden, kiln baking garden, and so on. Relying on the water resources of Yongjiang River, the town has built a bicycle riding area, equipped with coastal auxiliary facilities; at the same time, there are also water projects such as water motorboats. The town has held many time equestrian competitions, professional equestrian clubs, has built professional sports training bases, and embraces many sports and leisure facilities, such as vertical fishing, CS, and go kart. With its complete facilities and pleasant ecological environment, the town is not only a spring outing place for many colleges and universities, but also a high-frequency choice address for tourists.

The operation mode of the town is as follows: Sports + leisure + tourism. The planned areas include leisure sports area, water sports area, racecourse area, cultural block. The town is expected to have a good prospect due to its development status in all aspects. It is an industrial demonstration base in the province. The government has injected capital into it and completely planned a number of sports-related development plans, ecological protection plans, and public service plans to help the sustainable development of the town.

## 3. The Analysis and Research on the Development of Sports Characteristic Small Town in Guangxi

### 3.1. Analysis on the Development Characteristics of Sports Characteristic Small Town in Guangxi

It is connected with Guangdong, Yunnan, Guizhou, and Hunan, and the south is adjacent to the coast. The province is dominated by ethnic minorities, with a strong cultural atmosphere of ethnic minorities, a long history, and distinctive characteristics [15]. Because of its unique characteristic culture, it is an excellent help to build a characteristic town.

#### 3.1.1. Combination of Natural Resources and Social Security

Guangxi belongs to the subtropical monsoon climate region, with hilly terrain, surrounded by mountains, mild climate, and moderate temperature. Suitable for outdoor physical exercise, the call of corresponding countries in Guangxi to build sports characteristic town, documents have been issued to give policy support. Competent enterprises will invest and jointly practice the development and construction of small town with local people so as to make good use of the local mountains and rivers and reasonably develop them.

#### 3.1.2. Combination of National Characteristics and Sports Leisure

Guangxi Province has the largest ethnic population, including more than a dozen ethnic settlements composed of Zhuang, Yao, and Maonan. The resident population of Yao and Zhuang accounts for nearly 70% of the country. Because the cultural styles and characteristics of different ethnic minorities in China are different, and the historical cultural accumulation has a more Chinese flavor, the combination of ethnic style culture and sports characteristic small town can not only give full play to the characteristic culture and historical culture of ethnic minorities and help the wide dissemination of the unique culture of ethnic minorities, it also allows people to exercise with the unique sports of ethnic minorities, which not only promotes people's relaxation and entertainment, but also promotes the communication and integration of the civilizations of ethnic minorities [16, 17].

#### 3.1.3. Combination of Humanistic Care and Technical Support

Guangxi has a long history and culture since ancient times. Different ethnic minority residential areas have their unique folk characteristics. Clothing, food, and customs are different. In the past, due to its inconvenient transportation and less communication with the outside world, the traditional culture is well preserved; characteristic towns can take advantage of this cultural resource, integrate its culture into the construction of sports town, and form a comprehensive sports town with characteristic culture as the carrier and sports in it.

### 3.2. Comparative Analysis on the Development of Sports Characteristic Small Town in Guangxi

#### 3.2.1. Responding to the Policy and Strong Support from the State

Most of the sports characteristic small towns built in China respond to the national policy call and promote local economic development. Under the guidance and policy support of the local government, they assist the applicant enterprises to complete the implementation of the project, boost the forward development of society, provide jobs, improve the quality of life of local people so as to respond to the national policy, and boost the development of regional urban integration. It can be seen from Table 2 that the state supports and attaches importance to local society.

#### 3.2.2. Integration of Industry and City and Diversified Development

The construction of a sports featured town inevitably requires multi-industry cooperation to form an integrated ecological chain system. Relying on the terrain environment of the town and based on sports events, it drives the regional multi-industry development and makes up for many disadvantages of the development of a single industry, and the joint development of many businesses can radiate the common development of many surrounding businesses. While improving the employment rate, it also promotes the pace of urbanization and attracts sports lovers and tourists to visit.

#### 3.2.3. Thematic Development and Characteristic Material Selection

The core concept of the vigorous development of small town with Chinese sports and cultural characteristics is “characteristics,” that is, to “theme.” The establishment of small town with domestic sports and cultural characteristics is in full swing. If each small town does not have its own unique development “characteristics,” the construction is similar, thousands of articles are the same, and the architectural style and leisure mode are the same; it will inevitably lead to vicious competition of similar products. It is completely opposite to the original policy of designing and creating characteristic small town. The situation in each region is different. When designing a small town with sports characteristics, it needs to make rational use of local natural resources. In the design, reasonable layout is carried out around the construction theme to bring tourists a unique experience, especially outdoor lovers. They travel to experience different feelings. Therefore, in the design of the layout of the town, emphasis is placed on personalization and theme, with unique characteristic elements, and the characteristics of the town are fully described in terms of content, form, culture, and so on, Only then can we attract more tourists to travel and better promote the development of sports characteristic town.

#### 3.2.4. Green Construction and Rational Layout

The geographical environment and natural resources of each region are the source of its characteristic development, especially the areas with good natural environment protection and less environmental pollution are the first choice for the construction of characteristic small towns. With good environmental protection, the landscape planning of the small town can be carried out with the help of this characteristic to realize green economy.

When positioning the characteristic layout of the sports town, it determined the direction of its combined sports health industry, fully considered the natural environmental factors, such as area, location, shape, landform, wind direction, and sunshine conditions in the architectural design, made a reasonable plan for the feasibility and installation of its internal and external equipment and facilities, and made the layout of the park scientific, reasonable, and feasible, There are obvious sports areas, as well as activity areas for characteristic projects and derivative projects. The overall layout of the town is reasonable, feasible, and sustainable.

### 3.3. Analysis on the Development Trend of Sports Characteristic Small Town in Guangxi

#### 3.3.1. Analysis on the Advantages and Disadvantages of the Development of Sports Characteristic Small Town in Guangxi

The development of the region is inseparable from the strong support of the government. As shown in Table 3, it is the policy support of the government that makes the construction and development of small town with sports characteristics possible. Guangxi has superior geographical resources and many natural landscapes. Mashan County, Guangxi Province, relies on the terrain characteristics; it plays an important role in the development of small town. It can be seen from Table 4 that the small town has good resource advantages. It uses ecological resources to drive economic development and boost the development of the small town. From the data Table 5, except for the large number of participants in rock climbing competitions in Mashan County, the number of participants in competitions in other regions is relatively small compared with that in other parts of the county. The reason is that the publicity of the town is not in place, people's participation in the event is poor, and some events lack the calling ability.

#### 3.3.2. Development Trend Planning of Guangxi Sports Characteristic Town

Guangxi Province is expected to build 15 small town with sports characteristics. With the cooperation of enterprises and scenic spots, it will give full play to various advantages and characteristics and jointly improve its own and local economic strength. The development of a small town first needs smooth land transportation. The convenience of transportation directly affects the development prospect of the town. Secondly, the local unique national culture and customs have strong competitiveness. Therefore, its personalized characteristics should be fully reflected in the planning and then combined with the integrated development of multiple industries. With the help of various resource platforms, cooperate with upstream and downstream enterprises to build an ecological industrial chain, and finally plan a sustainable development construction plan for the future of the town on the basis of the above.

## 4. The Research on the Development Norms of Sports Characteristic Small Town in Guangxi

### 4.1. Normative Principles for the Development of Sports Characteristic Small Town in Guangxi

The standard principle is the cornerstone of the development of small town with sports characteristics. Reasonable standard regulations and scientific and reasonable standard principles play a key role in the construction of small town with sports characteristics.

#### 4.1.1. Principles of Promoting Sports Industry

Sports characteristic towns rely on sports events and combined with the common development of various industries, promote the accelerated development of local economy and promote the process of local urban integration construction. “Sports” itself cannot bring economic benefits, but the “sports +” mode can promote the common development of all sectors of society based on sports. The establishment of small town with sports characteristics is to take “sports” as the core foundation, combine diversified factors, integrate multiple industries, build an ecological chain, form a scene of common prosperity of multiple industries, and help the local economy take off.

#### 4.1.2. Principle of Promoting Residents' Health

One of the purposes of the state to advocate the construction of sports and health small town is to strengthen people's awareness of physical exercise. While sports characteristic small towns bring economic benefits to local people, they also publicize sports projects so that people all over the country can participate in sports and further improve people's physique. The current society is facing many problems, such as aging and frequent diseases, which also poses a heavy burden on social medical treatment. Therefore, the establishment of sports featured small town also increases people's enthusiasm for exercise and promotes people's health.

#### 4.1.3. Principle of Promoting Humanistic Harmony

Guangxi is a place dominated by ethnic minorities and has a strong historical and cultural atmosphere. With the laying of provincial, municipal, and county-level roads, the opportunities for ethnic minorities to communicate with the outside world have increased. The construction of sports green small town has driven the prosperity of local tourism and related industries. Tourists from all over the world can pass through small towns to have a better understanding of the national culture of the region so as to enhance historical and cultural exchanges among ethnic minorities. The combination of sports town and ethnic minority culture makes the local material and intangible cultural heritage well known to the world and promotes the development of ethnic minority culture and the establishment of unity and friendship among all ethnic groups.

### 4.2. Connotation of Development Norms of Sports Characteristic Small Towns in Guangxi

The standardized operation and management of small towns with sports characteristics is not only an important problem in their actual operation, but also the most direct experience for tourists. Its contents mainly include the rational use of natural resources, the construction of leisure infrastructure, the combined operation of multiple industries, social publicity and national characteristics, and ecological resource protection.

#### 4.2.1. Utilization of Natural Resources

The ecological natural resources in Guangxi are not only the support for the establishment of sports characteristic small town, but also the basic condition for their sustainable development in the future. When designing and planning the layout of the town, select appropriate areas scientifically and reasonably. The surrounding environment should be close to the city and close to the mountains and rivers. According to the characteristics of local mountains, plan appropriate sports events, fully combine with local geographical conditions and water resources conditions, and make use of and develop them to fully explore the advantages of local mountains, geography, or water resources.

#### 4.2.2. Social Mechanism Construction

It has also built sewage purification system, social security system, greening and emission reduction system, ecological environment system, health and safety system, and other aspects of small towns with sports characteristics in Guangxi so as to comprehensively coordinate the relationship between man and nature and the sustainable development of economy and society. It has brought valuable environmental protection heritage and suitable leisure sports environment to the construction of small towns with sports characteristics so as to effectively promote the long-term development of small towns. Do a good job in the work of the small town, adhere to the leadership of the local government and the input of all sectors of society, and establish and improve the small town-based health service network. Further improve the medical security level of sports villages and towns and share resources in the surrounding cities and towns where there is a lack of professional hospitals. It not only serves tourists, but also provides the best first-aid measures for the general public, personnel and fitness experiencers. Comprehensive services facilities and facilities with sports characteristics small town should be built.

#### 4.2.3. Characteristic Humanistic Management

The majority of ethnic minorities in Guangxi have rich cultural heritage. All ethnic groups have different ethnic cultural characteristics. In the past, the traffic was blocked, and the traditional culture was well preserved. Therefore, the original national culture has fresh vitality and attraction. The planning and design of the sports featured town combines the characteristics of national culture with sports, constructs the unique cultural characteristics of ethnic minority areas, and plans ethnic custom areas, folk custom museums, and other ways to let tourists know more about ethnic minority culture. By using high-tech means and buildings with national characteristics, tourists can experience the customs of ethnic minorities and create a small town with distinctive ethnic characteristics so as to attract more tourists.

### 4.3. Development Standard Design of Guangxi Sports Characteristic Town

The current construction and long-term development of sports characteristic small town need the continuous promotion of social forces and the integration of multi-industries and multifields for common development. Among them, the unique characteristics of small towns are the basic conditions for their initial planning and establishment, and the future sustainable development is the basic condition for their long-term operation.

#### 4.3.1. Characteristic Management

The characteristic construction mainly focuses on the further development of cultural projects and commodities with local ethnic characteristics in Guangxi so as to promote the vigorous development of small town with sports characteristics in Guangxi. Through construction, integrate the national characteristic commodity production line with product marketing services, promote local characteristic products, green environmental protection products, sports assembly R&D and sales in related industries, drive the upstream and downstream supply chain of production, emphasize multimode economic development, innovation, and upgrading, and manage market-oriented investment by integrating characteristic technologies of various industries, form a mutual aid economic development model with sports and related industries as the core industry, broaden their own industry characteristics, gradually develop to a multidimensional economy, and attract more private enterprises to invest in construction so as to produce the aggregation effect with sports as the core, increase the employment efficiency for the local, and promote the local economic and social development.

#### 4.3.2. Sustainable Development

In order to ensure the future sustainable development planning of the town, the plan is implemented from the following aspects:

*Science and Technology Publicity*. Use the current high-tech functional equipment to webcast all kinds of ethnic programs, competitions, and cultural activities held in the town through the webcast platform to attract network traffic and achieve the publicity effect. In addition, advertising can be carried out on video websites to attract people's attention so as to promote the town and attract tourists.

*Marketing*. Carry out business intervention on major tourism apps so that when browsing the web, people can also understand the characteristic town and facilitate business operation. Through the selected business promotion types, the majority of tourists can know more directly and clearly in advance. The business characteristics and project types of sports towns also increase their competitiveness when playing the effect of publicity and promotion and make them convenient for consumers. Carry out joint promotion with various organization types, such as travel agencies, so that the public can more effectively and directly understand the rich colors of small town with local sports characteristics, use various ways to enhance the popularity of small town, promote the development and growth of small town, and establish a perfect incentive mechanism for the sustainable development of small town.

*Ecological and Environmental Protection*. Science and greening are not only the characteristic signs of the town, but also the hot spots that people should pay attention to. Therefore, in the construction of the town, we must reasonably and actively protect the natural resources and promote the peaceful development of the environment and human society. Environmental awareness is the most fundamental, master environmental protection knowledge and cultivate environmental protection awareness, and take appropriate protection environmental measures and precautions against environmental problems. By doing a good job in publicizing the common sense of ecological and environmental protection for tourists in small town, this have gradually attracted people's attention to ecological and environmental problems. From the system, such as establishing an express sign, improving the legal system, doing a good job in the deduction and punishment performance evaluation system for environmental protection projects in small town, and gradually forming and improving the rules and regulations system, it provides a strong practical guarantee for the environmental protection of small town with sports characteristics so that small town with sports characteristics can coexist harmoniously with the natural environment and green and sustainable development.

### 4.4. Normative Effect of the Development of Sports Characteristic Towns in Guangxi

The construction of small towns with sports characteristics has promoted the integration and sound development of local sports, economy society, and humanities and science. After the overall normative construction and taking the normative effect as the empirical evaluation standard, it has effectively promoted the vigorous development of small towns with sports characteristics in China.

#### 4.4.1. Economic Promotion Effect

The establishment of the comprehensive economic development plan of Guangxi sports characteristic town can enhance the consumption resources of local industries and absorb more commercial enterprises and more diversified service industries. The good business environment promotes the vigorous development of market operation and increases many entrepreneurships and opportunities for local people so as to solve the economic development of some places and increase economic income. Thus, an upstream and downstream supply chain linked with sports has been formed. At the same time, it focuses on the multimode development of the industry and the improvement of technological innovation; through the integration of key technologies in various industries and market-oriented investment operation, a mutually beneficial economic development focusing on sport industry is formed, broadened its own industry characteristics, gradually developed into a multidimensional economy, and attracted more private enterprises to invest in construction. A gathering effect centered on sports has been formed, which has increased the employment efficiency of local people, further promoted social economic development and basically completed the construction and development of the national targeted poverty alleviation project.

#### 4.4.2. Humanistic Promotion Effect

For the local people, the construction of small town with sports and cultural characteristics can not only drive the vigorous development of local social, cultural, and economic industries, but also improve the local humanistic care. Let the traditional history, culture, and cultural customs of the town and its surrounding areas be understood by outsiders, and through the organic integration of local social material and cultural development, we can realize the mutual complementarity of the advantages of cultural resources, thus driving the sustainable development of social and cultural industries and the dissemination of cultural and historical products so as to improve the value performance of local cultural and social material heritage. It has enhanced the humanistic publicity value accumulated in the history of local ethnic groups, provided characteristic and personalized brand benefits for local culture, further improved the social awareness of the town, and indirectly promoted the local people to participate in the construction of their own national civilization by vigorously excavating the cultural brand value of their own national folk customs, historical life, material and nonmaterial civilization, further enhance the local people's recognition of their own humanistic values, further develop into a small town with sports characteristics rich in national cultural traditions, build and develop together with local humanistic values, and further improve the embodiment of local humanistic brand value.

## 5. Conclusion

The common features of the town are abundant resource advantages, prominent ethnic characteristics, strong cultural atmosphere, and support from local government departments, which have laid a foundation for the development of the town. From the eight sport characteristic towns studied, the scope roughly includes the following:

Natural sports characteristic town: Mashan County sport characteristic towns mainly focuses on rock climbing and mountaineering.

The small town with ethnic minority sports characteristics: Hechi Nandan Gayasi Valley sports characteristics town, it mainly performs ethnic minority competitive plays.

The town's leisure and sports culture features mainly fall into two categories: Fangchenggang sports features the town is mainly made up of sailing boats and motor boats on the water, and the beautiful south sports features the town is made up of fishing and kart competitions.

The subsidies of stadiums and gymnasiums have a strong locational effect on urban development [18], and the influence of marketing on host cities is strongly correlated with the exposure of sports events [19], so national sports organizations can strengthen the sponsorship of sports towns [20].

With the help of unique festivals, events, geographical location, natural environment, and other resource advantages, small town with sports and cultural characteristics in Guangxi will present the integrated development characteristics of multiple modes, such as “sports + vacation,” “sports + ethnic minorities,” and “sports + ecological resources,” which has laid a good, diversified foundation for the sustainable development of small town in the future. At the same time, the town pays attention to green ecological and environmental protection and the protection of the natural environment. It is believed that after scientific and reasonable design and layout, under the influence of some measures taken by the government and through continuous innovation and optimization, small town with sports characteristics in Guangxi will certainly obtain high-quality development and help promote the realization of the strategy of “healthy Guangxi 2030.”

## Figures and Tables

**Figure 1:** Research roadmap.

**Figure 2:** Rock climbing sports characteristic town in Mashan county.

**Figure 3:** Gayasi valley sports characteristic town.

**Figure 4:** Fangchenggang sports characteristic town in China.

**Table 1:** Names of eight sports featured small towns launched in Guangxi.

Declaration unit	Industrial orientation	Name of sports featured small town to be included in the cultivation list
Fangchenggang Heju real estate co., ltd.	Sports + industry + events	Fangchenggang sports townlets, China
Mashan county bureau of culture, press, publication, radio, television and sports	Sports + tourism + events + industry	Guling town, Mashan county rock climbing characteristic sports small town
Guangxi Dongmou tourism development co., ltd	Sports + tourism + folk custom	Gayasi valley leisure sports characteristic small town, Nandan county, Hechi
Xixiangtang district bureau of culture, press, publication and sports	Sports + leisure + tourism	Beautiful southern riding sports characteristic small town
Wen Xin Guang Ti bureau of Ziyuan county	Sports + tourism + culture	Chetian small township sports characteristic small town, Guilin resource county
Liuzhou Luzhai county sports bureau	Sports + culture + leisure	Zhongdu Shili Luojiang sports characteristic small town, Luzhai county, Liuzhou city
Guigang Guiping Xishanquan culture and sports bureau	Sports + tourism + health preservation	Guigang Guiping Xishanquan sports characteristic small town
Culture, radio, television, press, publication and sports bureau of Yizhou district, Hechi city	Sports + ecology + tourism	Hechi Desheng Lalang ecological leisure sports characteristic small town

**Table 2:** National policies on promoting sports construction and development.

Time	Department/name	Relevant content and purpose
December 2, 2016	“Guiding opinions of the general office of the state council on accelerating the development of fitness and sports industry”	It is planned to build 100 tourism demonstration bases with high influence, high popularity, and perfect service quality and agglomeration competitiveness in China. Driving large-scale mass tourism and a tourist destination for economic development

May 2017	Notice of the general administration of sports on promoting the construction of sports and leisure characteristic small town	Support the establishment of a small town with sports leisure and fitness cultural characteristics in China with prominent sports characteristics, strong cultural atmosphere, centralized integration of business forms, and superior natural environmental conditions and benefiting the physical and mental health of the general public

March 2018	“Guiding opinions of the general office of the state council on promoting the development of tourism in the whole region”	Promote the integrated development of national travel and sports, culture, education, science and health, vigorously develop travel services such as ice and snow sports, mountain outdoor sports, water sports, flight culture and scientific health Qigong education, reasonably develop idle space, venues and natural scenic spots, and integrate resources to form a cultural tourism complex

March 2019	The general administration of sports of the people's Republic of China issued the guidelines for the construction of pilot projects of sports and leisure characteristic small town	In China's central development area, adjacent to cities, regions, and other important hub areas with convenient transportation, we should promote the integrated development of tourism, exhibition, media, culture and entertainment based on sports, establish an innovative development system of “sports + ecosystem” and adjust measures to local conditions. Based on industry, conduct steady operation and innovative development, and actively build a national demonstration base for sustainable industrial construction

**Table 3:** Construction policies of small town with sports characteristics.

Particular year	File name	Relevant contents of sports town
June 1, 2017	“Healthy Guangxi 2030 plan”	Promote the comprehensive planning and construction of small town and the health of social people's livelihood and build a distinctive health preservation and leisure demonstration area. We have successfully held large-scale international activities and promoted the development of leisure, entertainment, and sports events

May 19, 2017	The 13th five-year plan for the development of housing and urban rural construction in Guangxi	Achieve scientific and reasonable urban and rural construction, perfect planning functions, and town construction into a unique village and town charm with prominent industrial development characteristics, beautiful environment, low-carbon life, perfect facilities, comprehensive services, democratic management and harmonious rural style, highlighting vitality, greenness, liveability, civilization, and happiness

October 30, 2018	Detailed rules for acceptance and evaluation in the cultivation stage of sports characteristic small town in Guangxi (for trial implementation)	The state will promote the construction of small town with sports and leisure characteristics and promote the sustainable development of small town with sports and leisure characteristics. Promote the in-depth integration and overall development of urban and rural national healthy cause and public hygiene under takings and health undertakings

July 28, 2017	The 13th five-year plan for the development of Guangxi sports industry	To build Guangxi brands, a number of sports industry bases were cultivated and the coordinated development of sports industry and cause was promoted

**Table 4:** Events held in Mashan county in the recent two years.

Date	Event name	Number of participants (PCs)
April 2018	Mashan county Yueyue ecological culture sports tourism festival Gu zero special event and “March 3” Shifeng Sihuang music festival and mountain motorcycle cross-country race	104
May 2018	China ASEAN rock climbing masters match	118
August 2018	National youth outdoor camp conference	470
October 2019	The 5th national junior rock climbing championship	320
October 2019	2019 Guangxi ring road cycling world tour (Mashan stage)	324
October 2019	China mountain marathon series 2019 China ASEAN mountain marathon and “run Guangxi” ecological marathon series (Mashan station)	690

**Table 5:** Combination of sports characteristic small town and scenic spots in Guangxi.

Name of sports featured town	Core scenic spot	Surrounding scenic spots
Characteristic town of rock-climbing sports in Guling town, Mashan county	Nothing	Lingyang temple, Jinlundong scenic spot, and Nongla nature reserve

Hechi south danger IELTS valley sports characteristic town	China Baiku Yao folk custom garden	

Fangchenggang sports characteristic town, China	Nothing	Xiwan tour scenic spot, Fangchenggang wetland park, Xiwan tour scenic spot, Yueliangwan scenic spot, and three-block-stone ocean park

Chetian small township sports characteristic town, Guilin resource county	Wupaihe drifting scenic spot	Guilin Zijiang scenic spot

Beautiful southern seven-star sports town	Old kapok carpenter's garden, phoenix garden, our courtyard, sun valley sports park, rose manor, Yicang Huahai scenic spot, etc.	QIPO forest farm Longtan point, Longmen Shuidu, Nanning zoo

Hechi Desheng Lalang leisure sports characteristic town	Panoramic view of Lalang ecological leisure tourism area and Lalang forest farm	Jinlangwan scenic spot and Huaiyuan ancient town scenic spot

Zhongdu Shili Luojiang sports characteristic town, Luzhai county, Liuzhou city	International 4A scenic spot	Xiangshui waterfall and Xiangqiao karst national Geopark in Zhongdu town

Guigang Guiping Xishanquan sports characteristic town	Nothing	Longtan national forest park, Guiping Xishan scenic attraction spot

## Data Availability

The experimental data used to support the findings of this study are available from the corresponding author upon request.
